The article "Curative Effect of Foraminal Endoscopic Surgery and Efficacy of the Wearable Lumbar Spine Protection Equipment in the Treatment of Lumbar Disc Herniation" was retracted in 2023. Reasons: signs of a paper mill; suspected computer-generated content; unreliable results or conclusions; lack of ethics approval or compliance.

# Curative Effect of Foraminal Endoscopic Surgery and Efficacy of the Wearable Lumbar Spine Protection Equipment in the Treatment of Lumbar Disc Herniation

**DOI:** 10.1155/2022/6463863

**Published:** 2022-03-25

**Authors:** ZhaoWu Meng, JinYang Zheng, Kai Fu, YiZhao Kang, Liang Wang

**Affiliations:** Sunshine Union Hospitai,Spinal Surgery, Weifang, Shandong 261000, China

## Abstract

Lumbar disc herniation is a common and frequently-occurring disease in pain clinics. The incidence rate of affliction is increasing with every passing year. Besides the aged, young people also suffer from long-term pain, which not only affects their daily routines but may also lead to serious impairment. The causes of chronic low back and leg pain caused by lumbar disc herniation are mainly related to mechanical compression, the adhesion of epidural space, intervertebral space, and aseptic inflammatory reaction. The treatment of lumbar disc herniation should follow the principle of step-by-step treatment. An appropriate treatment scheme needs to be adopted according to the patient's condition. About 80% of patients received nonsurgical treatment to get relief from the pain symptoms. However, 10% to 15% of patients still need traditional open surgery. Spinal foraminal surgery is a new method for the treatment of lumbar disc herniation, lumbar surgery failure syndrome, and lumbar spinal stenosis. However, there are only scattered clinical reports on the efficacy of spinal foraminal surgery. Based on it, this paper proposes a method to explore the efficacy of spinal foraminal mirror surgery in the treatment of lumbar disc herniation. Besides, postoperative wearable lumbar protective equipment is proposed to ensure a seamless rehabilitation effect on the patients. Statistical analysis performed using a *t*-test revealed that there was a significant difference between the visual analog scales (VAS) scores of the two groups after 3 and 6 months of treatment (*P* < 0.05). The paper analyzes and summarizes the cases with definite and poor curative effects, which not only provides the basis for clinical practice but also paves the way to multicenter clinical research.

## 1. Introduction

Pain is a signal of human body damage or disease invasion. Pain is considered one of the factors affecting the routine mode of living. It is also the main reason for patients to see a doctor and the main complaint of the first diagnosis. As a symptom, chronic pain has attracted great attention all over the world [1]. The world pain conference defined pain as “the fifth vital sign of mankind” after respiration, pulse, body temperature, and blood pressure. 80% of adults have experienced low back and leg pain. The incidence rate of lumbar disc herniation is 7.62% in China [2]. The proportion of surgical treatment for lumbar disc herniation in China has reached 0.12%. Likewise, the incidence rate of affliction is on the rise. The cost of treatment increases economic burdens and may lead to depression in patients and families. Anxiety and bad mood caused by pain seriously affect the work and life of patients [3].

The mechanism and etiology of lumbar disc herniation include the mechanical stimulation of nerve endings outside the fibrous ring, direct compression of nerve roots, and inflammatory stimulation induced by the compression of the nucleus pulposus [4]. It results in a series of symptoms, such as radiation pain. Other studies have shown that it is related to autoimmunity, smoking, gender, obesity, weight-bearing degree, and other factors. The treatment of lumbar disc herniation follows the principle of step-by-step treatment. Conservative treatment should be considered in the early stage [5]. If the formal treatment is ineffective or the symptoms are aggravated, minimally invasive treatment or open surgery should be considered. Of course, the surgical effect is the most accurate one. Because of the relatively large surgical incision, more muscle stripping and more bone tissue resection may destroy the stable structure of the spine. The treatment cycle of affliction is relatively long, which most of the patients find difficult to follow [6].

There are many surgical methods for the treatment of lumbar disc herniation, which can be summarized as traditional open surgery and minimally invasive surgery. The laminectomy and decompression of the nucleus pulposus with traditional open surgery is still a common surgical method in clinics. However, compared with minimally invasive surgery, open surgery causes greater trauma and damage to the posterior column of the spine [7]. Although the decompression range is larger than minimally invasive surgery, it can lead to nerve root adhesion. Because of the large wound and scar formation, the surgery takes a longer time in postoperative recovery, besides other complications [8]. With the progress of science and technology, the concept of minimally invasive surgery has been enhanced and has attracted the research community. Therefore, surgeons will have more consideration in the choice of surgical methods. With the rapid development and wider adaptation of technology, minimally invasive technology with less intraoperative and postoperative complications has become possible. With rapid postoperative recovery, little trauma, and less harm to spinal stability, minimally invasive technology is favored by surgeons and patients [9]. At the same time, with the continuous improvement of minimally invasive surgery technology, its scope of adaptation is also expanding, which can be well-applied to clinical practice. Hence, in recent years, minimally invasive surgery has been applied in clinics, and the promising results of the method have been reported in the treatment of lumbar disc herniation [10]. The schematic diagram of the lumbar intervertebral disc is shown in Figure 1.

Foraminal endoscopic surgery is a minimally invasive approach that preserves the multifidus muscle and delays the need for fusion. Unlike open surgery, the approach treats foraminal stenosis and requires only a small incision for the operation.

This paper presents a method to explore the curative effect of foraminal endoscopic surgery in the treatment of lumbar disc herniation. The original data are analyzed by the machine learning algorithm, and the curative effect analysis results are obtained. The research studies the wearable lumbar protective device after operation to further ensure the rehabilitation effect of the patients. Subsequently, the paper summarizes and analyzes the cases with definite and bad curative effects. The experimental results have laid a foundation for clinical research.

The remaining of the paper is organized into 5 sections.  Section 2 deals with the literature review. Details about the efficacy methods are presented in Section 3. The design and application of the wearable lumbar spine protection device are elaborated in Section 4. In Section 5, the experimental method is discussed with numerical findings and analysis. The last section, Section 6, is about the conclusion and future work.

## 2. Related Work

Low-back pain (LBP) is a prevailing affliction. It is reported that about 2 to 3 of adults suffer from LBP [11, 12]. The patients face difficulties to maintain healthy a lifestyle. According to [13], lumbar flexion and rotation are major causes of LBP. Though one of the main causes of LBP is lumbar disc herniation (LDH), 10-year research is necessary for the surgical approach to gain widespread popularity [14]. Details about the pain and treatment methods of LDH are discussed in the following subsections.

### 2.1. Research Status of Pain Mechanism of Lumbar Disc Herniation

Lumbar disc herniation is a low back and leg pain disease characterized by the degenerative changes of the lumbar disc, the rupture of the fibrous ring, the protrusion of the nucleus pulposus, and the stimulation or compression of the nerve root. Other causes include inflammatory reaction, low back pain, and radiation pain of the lower limb sciatic nerve under the action of external force [15]. The pain-causing mechanism of lumbar disc herniation is mainly related to the mechanical compression theory, inflammatory chemical stimulation theory, and autoimmune theory. The patient's bad mood, excessive body mass index, smoking, educational level, and blood circulation disorder may also be the causes of pain [16].

The theory of mechanical oppression comes first in the discussion of lumbar disc impairment. The lumbar intervertebral disc is composed of the fibrous ring and the nucleus pulposus. The fibrous ring is tough because of type I collagen. The nucleus pulposus has type II collagen and rich proteoglycan. Hence, it has good elasticity and fluidity under normal conditions. The prone lumbar segments are L4 ∼ 5 and L5 ∼ S1, accounting for more than 90% of the whole section. These two segments are located at the lumbosacral junction, with high mobility and high pressure [17]. Nerve root compression is the main cause of chronic pain in the lower limbs. As the spinal nerve root lacks the protection of the nerve sheath, slight compression will have obvious compression symptoms. With the extension of compression time, the normal metabolism of the nerve root is destroyed, and thus, the pain symptoms are obvious [18]. Yet, there is another theory, i.e., the theory of inflammatory chemical stimulation. Nerve roots compressed by the surrounding tissues are more likely to induce pain than the noncompressed nerve roots. Some nerve roots are not compressed. In such cases, patients have the symptoms of lower limb pain [19]. Oral nonsteroidal anti-inflammatory drugs or hormones can alleviate the pain, suggesting that chronic lower limb pain in patients with lumbar disc herniation is related to inflammatory response stimulation. This inflammation is not caused by pathogenic microorganisms like bacteria, however, aseptic inflammation is caused by ischemia or immunity. Long-term inflammation will inevitably produce fibrosis, leading to extensive tissue adhesion in the epidural space [20]. Finally, it is pertinent to discuss the immune response theory. The immune response theory of lumbar disc herniation holds that the extract of the intervertebral disc tissue has immunogenicity. Under normal circumstances, the nucleus pulposus tissue is wrapped in the annulus fibrosus. However, when the annulus fibrosus is broken, the nucleus pulposus protrudes from the disconnected position of the annulus fibrosus and even falls out of the annulus fibrosus [21]. The body considers the detached nucleus pulposus as “alien” and produces an immune response. The degree of immune response is positively correlated with the degree of the rupture of the annulus fibrosus and the prolapse of the nucleus pulposus [22]. The degree of pain is also related to the severity of the immune response. When the nerve without inflammation is simply compressed, its feeling and movement will be affected, however, there will be no pain. Only when the nerve with inflammatory stimulation is mechanically compressed, there will be pain. It can be seen that the autoimmune response plays an important role in chronic lower limb radiation pain [23]. The main factors of lumbar disc herniation are shown in Figure 2.

As observed in Figure 2, the main factors of low back and leg pain caused by lumbar disc herniation are mechanical compression, epidural adhesion, and inflammation. The compression of nerve roots plays an initiating role in the pain of patients with LDH, activating inflammatory chemical stimulation. Inflammatory stimulation leads to epidural adhesion, and epidural adhesion causes inflammatory stimulation and pain.

### 2.2. Research Status of Diagnostic Methods of Lumbar Disc Herniation

The diagnosis of the herniated lumbar disc (HLD) is rarely difficult and complicated. It can be diagnosed according to the patient's symptoms, positive signs, and imaging examination. Positive straight leg raise (SLR) test, sensory segmental pain, hypoesthesia, hyporeflexia or disappearance, and decreased muscle strength are some of the symptoms [24]. HLD can be diagnosed if three of the four criteria are met. The pain characteristics of HLD are as follows: the sensory changes and muscle strength changes of lower limb pain are consistent with the distribution characteristics of the nerve root segments. The cauda equina syndrome is an indication for immediate surgery. CT: in the past, it was considered that computed tomography (CT) was inferior to magnetic resonance imaging (MRI) in the diagnosis of HLD. CT discography can replace MRI in the diagnosis of lumbar disc herniation [25]. X-Ray film: it is a necessary examination for the diagnosis of HLD. It is recommended to give hyperextension and hyperflexion examination on the basis of frontal and lateral position to evaluate the stability of the lumbar spine.

Research shows that the results of CT and MRI are not positively correlated with the clinical symptoms of patients. Imaging suggests that the severity of HLD is serious; however, the pain symptoms of patients are not obvious, or there is no pain performance. Some patients have severe pain symptoms; however, the results of CT and MRI suggest that the severity of HLD is not obvious [26]. In [27], an SLR is performed to compare the efficacy of various treatment methods followed for lumbar disc herniation. The meta-analysis showed that lumbar discectomy LD is more effective than conservative care CC in treating herniation.

### 2.3. Treatment of Lumbar Disc Herniation

With the rapid development of China's economy and the popularization and improvement of medical insurance and rural cooperative medical care policies, people pay more attention to health. As a common disease, low back has attracted medical practitioners and researchers to treat low back and leg pain with a low cost and few side effects [28].

The early stage of HLD is mainly conservative treatment. It mainly includes bed rest, manual therapy, drug therapy, patient education, physical therapy, and nerve block. The traditional view is that bed rest is an effective treatment for both acute and chronic lumbar disc herniation. If conditions permit, they should be encouraged to go to the ground early. The curative effect of the patients is better than that of the nonexercise group. Patients with high exercise frequency and lower frequency of exercise have lower incidence rate of pain. Lumbar traction is effective in the treatment of sciatica [29]. The two methods can reduce the incidence of sciatica.

An epidural injection is a short-term outpatient operation, which can be carried out in doctors' clinics, hospitals, or surgical centers. It is highly effective and is a relatively safe and effective nonsurgical treatment option. One of the signs of success of epidural puncture depends on the sense of breakthrough. However, 30% of epidural puncture has no sense of the disappearance of resistance. Hence, imaging should be used to assist in positioning [30]. The needle entry path of epidural injection is carried out through the sacral hiatus approach, lamina space approach, and intervertebral foramen approach. The puncture through the sacral hiatus path is relatively easy to succeed and relatively safe. Its disadvantage is that the injection dose is the largest, usually 10 ml to 20 ml [31].

With the continuous development of clinical minimally invasive technology and the continuous improvement of imaging technology, the treatment of lumbar disc herniation is no exception. Clinicians pay more attention to minimally invasive treatment. Minimally invasive treatment methods are continuously improved [32]. Its advantages include small injury, fast postoperative recovery, and imaging guidance. Minimally invasive technology is suitable to accurately locate and improve the curative effect. Therefore, some patients can avoid the risk of open operation. Currently, minimally invasive treatment is performed through one or several small incisions through a percutaneous puncture or spinal endoscopy. Percutaneous transluminal endoscopic discectomy is a minimally invasive treatment that is widely used in clinical practice [33]. Surgical operation with microsystem has the advantages of short operation time, less intraoperative bleeding, rapid recovery, significantly shorter hospital stay, and higher pain relief rate of patients after hand surgery. The recurrence rate of postoperative pain within one year is between 2% and 10%. However, the technical route of the intervertebral foraminal mirror is steep, which has high requirements for the operator's technology, operating room machinery, and operating room environment [34]. A number of treatment approaches have been proposed so far in the literature. In the study [35], M. S. Kabil studied the far lateral lumbar disc herniation of 33 patients. The outcomes of the study suggest that the microendoscopic approach is safe and effective for treating back pain and lower limb symptoms. Waters et al. used the mathematical approach to estimate the LBP risks in manual lifting tasks [36], whereas assessed the risks factors involved in industries [37]. With EMG signals [38], the lumbar vertebrae pressure is computed during lying, sitting, and walking [39]. With lightweight bend sensors, Milea measured joint motion [40]. Some studies suggest the multimodal approach to treating LDH, including anti-inflammatory medications and physical therapy [41]. The research of Kim et al. compared the common treatments and preferred nerve injections [42] for affliction.

Tumor necrosis factor-alpha (TNF-*α*) is another widely used clinical treatment [43]. According to [44], TNF-*α* is effective in treating the sciatica of LDH patients. Intradiscal injection, however, has no benefit in such cases [45]. Thackeray et al. evaluated the profile of patients utilizing formal PT and their outcomes [46].

## 3. Efficacy Evaluation Method

This section, firstly, introduces the relevant theoretical knowledge of efficacy evaluation, and then the basic mathematical principle of support vector machine (SVM) is introduced. Following that, a method of efficacy evaluation of intervertebral foraminal endoscopic surgery for lumbar disc herniation based on SVM is discussed.

### 3.1. Correlation Theory

As a subjective discomfort, pain can usually clarify the location, nature, onset time, and inducement of pain. However, the severity of pain is an important reference index for assessing pain treatment. The key issue is how to measure subjective pain with objective indicators. Patients can evaluate themselves by representing different types of sensory scales. These methods are simple, feasible, and reliable. In clinical research, visual analog scales (VAS) are a measurement tool commonly used in pain assessment. However, the reliability of using it alone in pain research has been questioned by scholars. The Oswestry disability index (ODI) is a widely used low back pain evaluation index. The scoring table includes 10 observation items, including the degree of low back pain and leg pain, personal life and cooking, lifting heavy objects, walking, sitting, standing, sleeping, sexual life, social life, travel, etc. Each item is divided into 6 options from normal to abnormal, and the corresponding score of each option is from 0 to 5. Patients can choose according to their own situation and add the scores of 10 options. The calculation method of ODI score is given as follows:

(1) $$\begin{array}{c} \text{ODI}=\frac{\text{Actual Score}}{5\times \text{Number of questions answered}}\times 100\%. \end{array}$$

The lower the score percentage, the better the functional status, and the higher the score, the worse the functional status.

Patients' global impressions of change (PGIC) can reflect whether the patients' subjective pain is alleviated after the intervention of pain treatment. It can respond to the changes in the intensity and nature of subjective pain. It can also eliminate the patient's subjective misunderstanding that the reduction of pain is the improvement of the disease. According to the improvement of patients' condition, PGIC is divided into “1” for obvious improvement, “2” for slight improvement, “3” for no change, and “4″ for pain plus reuse. Patients with chronic low back and leg pain suffer from pain for a long time, and their work and life are affected to varying degrees. In the clinical study of chronic low back and leg pain, it is necessary to evaluate the changes of pain in combination with the patients' overall feeling and satisfaction with the treatment. The reason is that some research on the treatment of pain only aims to observe the changes of pain, however, it cannot treat the disease itself. Therefore, PGIC was selected as the evaluation standard for the efficacy of the two methods in the treatment of lumbar disc herniation. Then, the sample size estimation algorithm is introduced. Based on the difference test of two independent sample rates, the sample size calculation formula is as follows:

(2) $$\begin{array}{c} n_{1}=\frac{{\left[Z_{1-a/s}\sqrt{\bar{\pi }\left(1-\bar{\pi }\right)\left(1+1/\gamma \right)+Z_{1-\beta \sqrt{\pi_{1}\left(1-\pi_{1}\right)+\pi_{2}/\gamma \left(1-\pi_{2}\right)}}}\right]}^{2}}{{\left(\pi_{1}-\pi_{2}\right)}^{2}/\gamma }. \end{array}$$

Among them, *γ* is the proportion of the sample size of the two groups, *n*_1_ : *n*_2_=*γ*. $\bar{\pi }$ is the weighted average rate of two samples, and *π*_1_ and *π*_2_ are the two population rates, respectively. *Z* is the normal distribution. The research flow of the experiment is shown in Figure 3.

SPSS 21.0 was used for the statistical analysis of data. The measurement data are expressed by mean and standard deviation. The general data of the two groups were analyzed by chi-square test and analysis of variance. Paired *t*-test was used for intragroup comparison. Two independent sample *t*-tests were used for comparison between groups. The other measurement data were compared between groups by an independent sample *t*-test. The chi-square test was used to compare the gender composition ratio. The proportion of ineffective cases decreased the muscle strength, and hypoesthesia in the ENP group was tested by Fisher's exact test. The proportion of ineffective cases decreased the muscle strength, and hypoesthesia in the TFSI group was tested by approximate chi-square test. The test levels were all *P* < 0.05, with a statistical difference.

### 3.2. Efficacy Evaluation Method Based on SVM

The development of SVM theory is relatively mature. The SVM theory minimizes structural risk. Moreover, it can take into account the training ability and generalization ability. Moreover, it has very obvious advantages in solving the problems of nonlinearity, local minimum, small samples, and high dimension. It can be said that support vector machine provides a basic framework for machine learning. The basic principle of SVM is depicted in Figure 4.

When extending linear SVM to nonlinear SVM, we need to extend the linear partition to a general linear partition. Set the original training set as follows:

(3) $$\begin{array}{c} T=\left\{\left(x_{i},y_{i}\right),\left(i=1,2,\ldots ,l\right)\right\}\in {\left(R^{n}\times y\right)}^{l}. \end{array}$$

Then, spatial transformation is introduced, which is given as

(4) $$\begin{array}{c} \Phi :R^{n}⟶H,\\ x⟶z=\Phi \left(x\right). \end{array}$$

After transformation, the training set *T* becomes

(5) $$\begin{array}{c} T_{\Phi }=\left\{\left(z_{i},y_{i}\right),\left(i=1,2,\ldots ,l\right)\right\}\in {\left(H\times y\right)}^{l}. \end{array}$$

The linear partition hyperplane is finding out in the space. Next, the partition hypersurface and decision function on the original space are derived.

(6) $$\begin{array}{c} f\left(x\right)=\mathrm{sgn}\left(\left(w^{*}\cdot z\right)+b^{*}\right)\\ =\mathrm{sgn}\left(\left(w^{*}\cdot \Phi \left(x\right)\right)+b^{*}\right). \end{array}$$

It is noted that the distance between two hyperplanes in Hilbert space can still be expressed as *w*^*∗*^, which can be obtained as

(7) $$\begin{array}{c} \underset{w,b,\xi }{\min}\frac{1}{2}{\left\|w\right\|}^{2}+C\sum_{i=1}^{l}\xi_{i}\\ \text{s.t.}y_{i}\left(\left(w\cdot \Phi \left(x_{i}\right)\right)+b\right)\geq 1-\xi_{i},\;i=1,2,\ldots ,l\\ \xi_{i}\geq 0,\;i=1,2,\ldots ,l. \end{array}$$

In the above formula, *w* is the vector weight, while *C* and *ξ*_*i*_ are the penalty coefficient and relaxation variable, respectively. Introduce the Lagrange function.

(8) $$\begin{array}{c} L\left(w,b,\xi ,\alpha ,\beta \right)=\frac{1}{2}\;{\left\|w\right\|}^{2}+C\sum_{i=1}^{l}\xi_{i}-\sum_{i=1}^{l}\alpha_{i}\left(\left(y_{i}\left(w\cdot \Phi \left(x_{i}\right)\right)+b\right)-1+\xi_{i}\right)-\sum_{i=1}^{l}\beta_{i}\xi_{i}. \end{array}$$

For support vector machine, the kernel function is the key factor. Different kernel functions and selected parameters can affect the performance of support vector machine. For the theoretical research of support vector machine and for the application of SVM, the selection of kernel function and its parameters are particularly important. At present, among all classification algorithms, the most advanced is the kernel function method. The kernel function of SVM performs well in solving classification problems. In the selection of kernel function, there are two specific parts: one is to select the specific type of kernel function and the other is to select relevant parameters. Therefore, in the application field of SVM, one of the difficult problems is how to select the appropriate kernel function parameters according to the specific problems, which is also the focus of researchers. However, so far, there is no theory to guide the development of these two aspects.

In the field of kernel method, kernel function plays a very important role, which can effectively resolve nonlinearity and overcome the disaster of dimension. This part will focus on the basic properties and characteristics of kernel function. It is important in the construction of new kernel function and the implementation of SVM algorithm. A hybrid kernel function method is proposed, which can improve the performance of SVM. The form of hybrid kernel function is usually written as follows:

(9) $$\begin{array}{c} K_{\text{mixed}}\left(x,x^{\prime }\right)=\sum_{i=1}^{n}\rho_{i}K_{i}\left(x,x^{\prime }\right). \end{array}$$

where *n* refers to the weight of *n* different kernel functions, *ρ*_*i*_ is the weight, which refers to the weight of the *i*^th^ kernel function, and *K*_*i*_(*x*, *x*′) is the mixed kernel function. According to the kernel function theory, the mixed kernel function satisfies the Mercer condition. The kernel function constructed by the combination of different types of kernel functions can take into account the characteristics of its basic kernel function. In addition, the performance can be improved by adjusting the model parameters. To sum up, it can be considered to use the kernel function with strong generalization ability and the kernel function with strong learning ability for linear weighting to construct the hybrid kernel SVM algorithm. The combination of polynomial kernel function and sigmoid kernel function can theoretically improve the generalization ability and learning ability of SVM. The constructed hybrid kernel function has the characteristics of the above two basic kernel functions. Under some conditions, the properties of the sigmoid kernel function and RBF function are similar.

After normalizing the data, it is used as input data. Finally, the form of the mixed kernel function, the value range of parameters, and the method of parameter optimization are determined. The polynomial kernel with strong generalization ability and sigmoid kernel with strong learning ability are linearly weighted to construct the mixed kernel functioned SVM. In the training model, the grid search algorithm is used to optimize the parameters of the hybrid kernel SVM algorithm. Finally, the constructed hybrid kernel SVM algorithm is applied to the pulmonary nodule recognition to improve the accuracy and sensitivity of pulmonary nodule recognition.

## 4. Wearable Lumbar Spine Protection Device

After comprehensively comparing the existing equipment at home and abroad, it is found that almost all traction equipment cannot carry out lumbar push massage. A number of such devices have been designed with varying intrinsic issues. The device of extensible sensors is proposed by [47] to monitor lumbar flexion and rotation and to help diagnosticians in assessing the risk of low-back pain. However, because of the cumbersome setup, the device has wearability issues. Similarly, the inertial measurement unit (IMU) has also been utilized for measuring body motions [48]. Similarly, the inexpensive bend sensors-based equipment of [40] fails to detect three-axis motions of the lumbar joints. The lumbar-motion monitoring tool of [49] is heavy enough to be worn for a long time. The combined treatment scheme of traction and lumbar push cannot be realized. Therefore, this paper introduces the designs of a lumbar pushing traction treatment device that uses the combination of motor and hydraulic pressure to complete the treatment of the combination of traction and lumbar pushing. With the cooperation of a multisensor, it can realize the accurate control of traction force, traction distance angle, amplitude, and frequency of the push massage. The tool supports the cooperative treatment of push and traction. Moreover, the modular design and software design of the control system of the lumbar pushing traction treatment device is introduced. The effectiveness of the control system is proved by a prototype test. The overall results of the lumbar spine protection device are shown in Figure 5.

The lumbar pushing and traction device is a rehabilitation training system for the treatment of lumbar diseases. The device decomposes the lumbar back extension method, lumbar oblique pulling method, and pelvic traction method in massage manipulation into five actions: longitudinal traction, left and right rotation, left and right swing angle, up and down angle, and lumbar pushing and massage. The device design is mainly divided into the head chest plate and hip leg plate. The waist pushing device is located near the hip leg plate of the head chest plate. The whole bed can be pulled longitudinally, rotated left and right, swung left and right, and angled up and down.

The hydraulic system of the lumbar pushing traction treatment device is mainly composed of power components, executive components, control components, auxiliary components, and hydraulic oil. The power element adopts an internal gear pump, which can convert the mechanical energy output by the motor into liquid pressure energy, with low noise and high efficiency. The actuating elements include hydraulic cylinders and a hydraulic motor. The hydraulic cylinder is used to cooperate with the mechanical structure to drive the bed movement. The control components are various hydraulic valves, including directional valve, overflow valve, proportional valve, and one-way valve. With this setup, it becomes quite feasible to control and regulate the flow, pressure, and direction of liquid in the system. The lumbar pushing traction treatment device needs to complete longitudinal traction, left and right swing angle, left and right rotation, up and down angle, and lumbar pushing massage. To ensure the stability and safety of the system operation, the control system adopts the idea of modular design. The system is mainly composed of a power module, waist pushing module, traction module, and human-computer interaction module. The treatment posture is shown in Figure 6.

To realize the adjustable frequency and amplitude of waist pushing, it is necessary to control the speed of the DC motor and the displacement of the other two motors driving the mechanism. The speed of a DC motor determines the frequency of lumbar pushing, and the displacement of the motor mechanism determines the amplitude of lumbar pushing. By controlling two DC motors at the same time, the alternating movement or joint movement of two waist pushing mechanisms can be realized. In the process of lumbar pushing massage, aiming at the control problems of the left and right pushing devices, the system uses the PWM voltage regulation method to change the voltage of the two DC motors. Moreover, the system supports effortless changes in the speed of the motor through voltage regulation and alterations in the lumbar pushing frequency and realizes the adjustable lumbar pushing frequency.

## 5. Experiments and Results

To systematically evaluate the proposed approach, data about the patients suffering from LDH was collected and analyzed. Details about the experimental setup and analysis are discussed in the following subsections.

### 5.1. Relevant Preparations for the Experiment

Patients with lumbar disc herniation (LDH) were recruited from the pain clinic of the Department of Anesthesiology of Hospital. This study followed the requirements and principles of clinical research. The subjects were completely voluntary, and the information was kept confidential. After the study, privacy-related information was deleted from the patient's name, gender, age, ID number, and so on. Patients were kept unaware of the treatment cycle and general process to reduce their fear of treatment and enhance their confidence in treatment. Patients were demonstrated to correctly use the pain assessment scale for pain scoring.

After the first injection, the patients who received epidural injection through the intervertebral foramen reported that the pain relief was less than 50%. The patients were suggested to avoid taking painkillers, strenuous activities, and exercises that aggravate the load on the waist during treatment. As shown in Table 1, there is no statistically significant difference in gender, age, body mass index, and course of disease between the ENP group and TFSI group. It implies that the data of the two groups meet the requirements of clinical research, and the test data are comparable, as shown in Table 1.

Similar to the impact of demographic information on body weight and obesity [50, 51], there are different opinions on the influence of gender, age, weight, occupation, and other factors on pain score. Compared with other data, the *p* value is closer to 0.05. We further analyze the body mass index (BMI) and gender of the two groups to determine whether the BMI and gender have an impact on the pain score of the two groups in this study. BMI is a number obtained by dividing the weight in kilograms by the square of the height in meters. BMI is a neutral and reliable indicator. The BMI index of the domestic population is different from that of other countries in Europe and the United States.  Table 2 shows the changes of the VAS scores of BMI within and beyond the normal range in the ENP group before and after treatment.

Table 2 shows the changes in the VAS scores of BMI within and beyond the normal range in the ENP group before and after treatment. The VAS scores at each follow-up point after treatment were lower than those before treatment. The VAS score at each time point after treatment was compared between the groups. After the *t*-test, the results showed that there was no statistical significance between the groups (*P* > 0.05). In the TFSI group, whether BMI was within the normal range or beyond the normal range, it was improved compared with the same group before treatment. For the intergroup comparison, the VAS scores of the two groups before treatment, 1 month after treatment, 3 months after treatment, and 6 months after treatment were tested by the *t*-test for the two independent samples. The results showed that the difference was not statistically significant.

### 5.2. Experimental Result and Analysis

The intergroup comparison revealed that there was no significant difference between the two groups after treatment (*P* > 0.05). There was a significant difference between the two groups after 3 months of the treatment (*P* < 0.05). The VAS score of the ENP group was lower than that of the TFSI group. Six months after treatment, there was a significant difference between the two groups (*P* < 0.05). The VAS score of the ENP group was lower than that of the TFSI group. The VAS score changes of the two groups before and after treatment and at each follow-up point are shown in Figure 7.

The figure shows the change trend of VAS in the two groups at each follow-up time point before and after treatment. There was a significant difference between the two groups at three and six months after treatment (*P* < 0.05). Over time, the VAS score of the ENP group was lower than that of the TFSI group. Two independent sample *t*-tests showed that there was no significant difference in VAS between the two groups after treatment (*P* > 0.05). The changes of VAS between the two groups, 3 months, and 6 months after the treatment showed that the change range of the ENP group was significantly higher than that of the TFSI group (all *P* < 0.05).  Table 3 shows the changes in the number of people in the ENP group and TFSI group before, after, and at each follow-up time point compared with before treatment. It makes a comparative analysis between the groups, as illustrated in the table.

It is clear from Table 3 that there is no change in VAS in the TFSI and ENP groups after one month of treatment. No significant difference was reported between the two groups. The table also shows that there is no significant difference between the two groups in patients whose VAS score decreases ≥ 2 cm at one time after treatment. The comparison of the number of patients with VAS reduction ≥ 2 cm 1 month after treatment is shown in Figure 8.

It was observed that after treatment, the VAS pain score of the two groups decreased significantly as compared with that before treatment. The VAS score of the ENP group decreased more significantly than that of the TFSI group at 3 and 6 months of the follow-up. After treatment, the ODI scores of the two groups were significantly lower than those before the treatment. At 1 month, 3 months, and 6 months after treatment, the ODI value of the ENP group was lower than that of the TFSI group. During the whole study, two patients temporarily stopped treatment because they could not cooperate with local surgery. One patient complained of dizziness and nausea during treatment. After adjusting body position and fluid, the symptoms were relieved. However, the other patients had no adverse reactions.

## 6. Conclusion and Future Work

At present, domestic and foreign scholars are still exploring the influencing factors of intraoperative and postoperative complications of the efficacy of percutaneous transformational endoscopic discectomy (PTED) in the treatment of lumbar disc herniation. Combined with the experience of our department in PTED surgery, it is suggested that doctors who are about to carry out intervertebral foraminal endoscopy should have rich experience in open surgery and solid anatomical knowledge. The physician, on the basis of formal training, should gradually expand the indications of surgery. Initially, the main goal should be clinical efficacy with fewer complications. At present, local anesthesia is still the main anesthesia method for PTED. After accumulating rich clinical experience, our department found that general anesthesia is a feasible anesthesia method through a clinical test in the interlaminar approach. Local anesthesia combined with intravenous anesthesia can be selected in the lateral approach to reduce patients' pain and improve pain tolerance. In the current era of technology, medical surgery ought to make full use of the development of science and technology. The cutting edge-research studies suggest that spine surgeons should follow evidence-based medicine besides the concept of minimally invasive surgery. Moreover, as PTED has broader development prospects, the approach needs to be adopted to serve the human race in the best possible way. In this perspective, this research work proposes a method to explore the curative effect of foraminal endoscopic surgery in the treatment of lumbar disc herniation. The SVM machine learning classifier is utilized for the analysis of the curative effect. The findings of the experimentation reveal that the VAS pain score of the two groups decreases significantly after treatment. Moreover, it was observed that the ODI scores of the two groups were significantly lower than those before the treatment. Besides, this research work suggests the use of the wearable lumbar protective device for the effective rehabilitation of patients. To the authors' knowledge, this study is the first of its kind to apply ENP technology in treating HLD in China. Although the research is single-centered with a small sample, it provides preliminary, reliable, and scientific experimental data for the further study of ENP in the treatment of HLD.

This study is not free from limitations. The research targets only a follow-up of six months after the operation. After six months of pain relief, it is not known whether the patients treated with ENP will form epidural adhesion again. The research at this stage is quiet on such questions. In the future, we are planning to use other machine learning classifiers and a hybrid approach to further enhance the research work. Moreover, we look forward to the results of multicenter and large sample studies to further confirm the clinical significance of ENP in the treatment of HLD-derived chronic low back and leg pain [52].

## Figures and Tables

**Figure 1:** Schematic diagram of the lumbar intervertebral disc.

**Figure 2:** The main factors of lumbar disc herniation.

**Figure 3:** Research flow chart of experiment.

**Figure 4:** Basic principle diagram of support vector machine.

**Figure 5:** Overall structure diagram of lumbar protection equipment.

**Figure 6:** Treatment posture diagram of lumbar spine protection equipment after lying down.

**Figure 7:** VAS score changes of the two groups before and after treatment.

**Figure 8:** Comparison of patients with VAS reduction ≥ 2 cm 1 month after treatment.

**Table 1:** General information of two groups of patients.

Observation items	ENP	TFSI	T	*P*
Gender	15/12	23/28	0.773	0.379
Age	51.07 ± 16.13	47.78 ± 15.15	0.892	0.375
Body mass index	23.61 ± 1.81	22.93 ± 1.44	1.799	0.076
Course of disease	9.52 ± 5.65	8.84 ± 4.61	0.573	0.569

**Table 2:** Effect of BMI on VAS score.

Time	ENP			TFSI		
	BMI	T	*P*	BMI	T	*P*
Zero	5.36 ± 1.03	0.918	0.368	5.81 ± 1.38	0.757	0.453
One	2.09 ± 1.04	0.828	0.415	2.56 ± 1.67	0.883	0.382
Three	2.09 ± 1.14	0.384	0.704	2.25 ± 1.00	0.112	0.911
Six	2.82 ± 1.60	0.010	0.992	2.81 ± 1.42	0.031	0.975

**Table 3:** Comparison results of the proportion of people with changes in the VAS score.

Time	Unchanged		Rise		Reduce	
	TFSI	ENP	TFSI	ENP	TFSI	ENP
1 month	1 (51)	0 (27)	0 (51)	1 (27)	38 (51)	18 (27)
3 months	5 (51)	1 (27)	0 (51)	0 (27)	27 (51)	21 (27)
6 months	7 (15)	3 (27)	2 (15)	0 (27)	15 (15)	15 (27)

## Data Availability

The datasets used during the current study are available from the corresponding author on reasonable request.
